# AdaCN: An Adaptive Cubic Newton Method for Nonconvex Stochastic Optimization

**DOI:** 10.1155/2021/5790608

**Published:** 2021-11-10

**Authors:** Yan Liu, Maojun Zhang, Zhiwei Zhong, Xiangrong Zeng

**Affiliations:** School of Systems Engineering, National University of Defense Technology, Changsha 410073, China

## Abstract

In this work, we introduce AdaCN, a novel adaptive cubic Newton method for nonconvex stochastic optimization. AdaCN dynamically captures the curvature of the loss landscape by diagonally approximated Hessian plus the norm of difference between previous two estimates. It only requires at most first order gradients and updates with linear complexity for both time and memory. In order to reduce the variance introduced by the stochastic nature of the problem, AdaCN hires the first and second moment to implement and exponential moving average on iteratively updated stochastic gradients and approximated stochastic Hessians, respectively. We validate AdaCN in extensive experiments, showing that it outperforms other stochastic first order methods (including SGD, Adam, and AdaBound) and stochastic quasi-Newton method (i.e., Apollo), in terms of both convergence speed and generalization performance.

## 1. Introduction

Stochastic gradient descent (SGD) [1] is the workhorse method for nonconvex stochastic optimization in machine learning, particularly for training deep neural networks (DNNs). During the last decades, many accelerated first order variants of SGD are widely used due to their simplicity and versatility, including the accelerated SGD (ASGD) methods using Nesterov scheme [2], momentum [3] and heavy-ball method [4], and the adaptive methods such as AdaGrad [5], AdaDelta [6], RMSProp [7], and Adam [8]. Recently, Adam has become the default optimization method for many deep learning applications because of its rapid convergence speed and relatively insensitive choices of hyperparameters [9], and it also has engendered an ever-growing list of modifications, such as AdamW [10], NosAdam [11], AMSGrad [12], AdaBound [13], Radam [14], Sadam [15], and Adax [16], to name a few. The main difference between the ASGD methods and the adaptive methods is the former scales the gradients in different directions uniformly while the latter uses adaptively element-wisely scaled learning rates, which usually causes that the latter is able to converge faster and less sensitive to the learning rate than the former. However, it has been observed that the adaptive methods may converge to bad/suspicious local optima, leading to worse generalization ability than the ASGD methods [17], or fail to converge because of unstable and extreme learning rates [13].

The abovementioned methods, belonging to the stochastic first order method family, only use gradient information and do not consider the curvature of the loss landscape, thereby leading to their suboptimal behavior in algorithmic iterations. Instead, existing stochastic second order methods can capture and exploit the curvature properties of the loss landscape by incorporating both gradient and Hessian information. For example, stochastic Newton methods are typical ones that adopt exact stochastic Hessians. However, computing the full Hessian for training large-scale DNNs is prohibitively expensive, and thus it is necessary to approximate it or avoid directly computing it in algorithmic iterations. According to the way of approximating the stochastic Hessian matrix, stochastic second order methods for training large-scale DNNs can be broadly categorized into two branches: the stochastic quasi-Newton (SQN) methods approximate the Hessian as a series sum of first order information from prior iterations, such as AdaQN [18], SdLBFGS [19], and Apollo [20]; the stochastic second order Hessian-free methods compute the Hessian-vector product exactly through an efficient procedure proposed in [21], such as AdaHessian [22] which approximates the Hessian diagonal using Hutchinson's method based on the Hessian-vector product, which is significantly more costly than SQN methods.

Recently, based on a classic method in the nonstochastic setting, the cubic regularized Newton method [23], the stochastic adaptive regularization methods using cubics (SARC) [24–26] are proposed to address relatively small-scale nonconvex stochastic optimization problems, and they find the minimizer of a local second order Taylor approximation with a cubic regularization term at each iteration. It is observed that the SARC methods are able to escape saddle points more efficiently, leading to better generalization performance than most of the abovementioned stochastic first order and second order methods [23, 27] in relatively small-scale machine learning problems. More recently, a variant of SARC combining with negative curvature (SANC) is proposed in [28] with even better generalizability since a direction of negative curvature also benefits escaping strict saddle points [29, 30]. Unlike previous SARC methods, the SANC uses independent sets of data points of consistent size over all iterations to attain stochastic gradient and Hessian estimators, making it more practical than SARC. However, SARC and SANC use a Krylov subspace method to iteratively solve a cubic regularized Newton subproblem and use a trust region-like scheme to determine if an iteration is successful or not and update only when it is successful, which hinders their applications in large-scale nonconvex stochastic optimization (in the sense of large datasets and/or high-dimensional parameter spaces). Therefore, these existing cubic regularized Newton methods are not suitable for training large-scale DNNs.

In this work, we develop a novel adaptive cubic Newton method, AdaCN, for large-scale nonconvex stochastic optimization, and it can inherit the superiority of SARC and SANC methods (i.e., great generalizability), but tackle their aforementioned challenges (i.e., unsuitable for training large-scale DNNs). AdaCN is designed for nonconvex stochastic optimization through dynamically capturing the curvature of the loss function by diagonally approximated Hessian and the norm of difference between previous two estimates. It only requires at most first order gradients and updates with linear complexity for both time and memory, thus it is quite suitable for large-scale nonconvex stochastic optimization problems. In order to reduce the variance introduced by the stochastic nature of the problem, AdaCN hires the first and second moment to implement an exponential moving average on iteratively calculated gradients and approximated Hessians, respectively. Therefore, these moments are able to not only accelerate convergence speed but also smooth the noisy curvature information and get an approximation to the global curvature information, avoiding misleading local gradient and Hessian information which can be catastrophic. The superiority of AdaCN can be illustrated with two simple 2D functions (one is convex and the other is nonconvex, and these two functions give hints to local behavior of optimizers in deep learning), as shown in Figure 1, where we show the trajectories of different optimizers. As can be seen, AdaCN can converge much faster than stochastic first order methods such as SGD and Adam and stochastic quasi-Newton method Apollo. Furthermore, we will experimentally show the superiority of AdaCN through image classification tasks: LeNet [31] on Mnist and VGG11 [32], ResNet34 [33], and DenseNet121 [34] on CIFAR10 and CIFAR100 [35] dataset; and language modeling task: LSTM [36] on Penn Treebank [37] dataset.

Notation: we use italics letters *α*, *β* to denote scalars, bold lowercase letters **x**, **y** to denote vectors, and bold uppercase letters **A**, **B** to denote matrices. For vectors, we use ‖·‖ to denote the *l*2-norm.

## 2. Formulation of Adaptive Cubic Newton Method

### 2.1. Problem Statement

In this paper, we consider the following stochastic optimization problem:

(1) $$\begin{array}{c} \underset{x\in {\mathbb{R}}^{d}}{\min}f\left(x\right)=E_{\xi ∼D}\left[f\left(x;\xi \right)\right], \end{array}$$

where *f* is a continuously differentiable function and possibly nonconvex, **x** ∈ *ℝ*^*d*^ is the parameter to be optimized, and *E* denotes the expectation with respect to **x**, a random variable with the distribution *𝒟*. A special case of (1) that arises frequently in supervised machine learning is the empirical risk minimization (ERM) problem [38]:

(2) $$\begin{array}{c} \underset{x\in {\mathbb{R}}^{d}}{\min}f\left(x\right)=\frac{1}{n}\sum_{i=1}^{n}f_{i}\left(x;\xi_{i}\right), \end{array}$$

where *f*_*i*_ : *ℝ*^*d*^⟶*ℝ* is the loss function corresponding to the *i*-th data instance, and *n* is the number of data samples that is assumed to be extremely large.

### 2.2. Newton Update from Cubically Regularized Model

We begin with a stochastic Newton (SN) method. At a high level, we sample two independent mini-batches *S*_*g*_ and *S*_*B*_ at each iteration, and the stochastic gradient and Hessian estimators, say, **g**_*k*_ and **B**_*k*_, can be defined as

(3) $$\begin{array}{c} g_{k}=\frac{1}{\left|S_{g}\right|}\sum_{i\in S_{g}}\nabla f_{i}\left(x;\xi_{i}\right),\\ B_{k}=\frac{1}{\left|S_{B}\right|}\sum_{i\in S_{B}}\nabla^{2}f_{i}\left(x;\xi_{i}\right). \end{array}$$

In each iteration of the SN method, gradient descent finds the minimizer of a local second order Taylor expansion

(4) $$\begin{array}{c} x_{k+1}=\underset{x}{\arg\min}f\left(x_{k}\right)+g_{k}^{T}\left(x-x_{k}\right)+\frac{1}{2}{\left(x-x_{k}\right)}^{T}B_{k}\left(x-x_{k}\right), \end{array}$$

and its corresponding Newton update is shown as

(5) $$\begin{array}{c} x_{k+1}=x_{k}-B_{k}^{-1}g_{k}. \end{array}$$

For large-scale stochastic optimization problems, the stochastic Hessian **B**_*k*_ is properly approximated. For example, AdaQN [18], SdLBFGS [19], and Apollo [20] (belonging to stochastic quasi-Newton methods) approximate **B**_*k*_ as a series sum of first order information from prior iterations, while AdaHessian [22] (one of the stochastic second order Hessian-free methods) approximates the Hessian diagonal using Hutchinson's method [39] based on the Hessian-vector product.

A new principled variant of the SN method that could enjoy global convergence guarantees is proposed in [23], and it finds the minimizer of the following cubically regularized second order approximation of *f* with **g**_*k*_, **B**_*k*_ and a sufficient large *ρ* > 0:

(6) $$\begin{array}{c} x_{k+1}=\underset{x}{\arg\min}f\left(x_{k}\right)+g_{k}^{T}\left(x-x_{k}\right)+\frac{1}{2}{\left(x-x_{k}\right)}^{T}B_{k}\left(x-x_{k}\right)+\frac{\rho }{6}{\left\|x-x_{k}\right\|}^{3}, \end{array}$$

where **x**_*k*_ is the value at *k*-th iteration. By first order optimality conditions, we set the derivative of the objective to zero, which immediately yields

(7) $$\begin{array}{c} g_{k}+B_{k}\left(x-x_{k}\right)+\frac{\rho }{2}\left\|x-x_{k}\right\|\left(x-x_{k}\right)=0, \end{array}$$

which is a nonlinear system and can be approximated by a linear one as follows:

(8) $$\begin{array}{c} g_{k}+B_{k}\left(x-x_{k}\right)+\frac{\rho }{2}\left\|x_{k}-x_{k-1}\right\|\left(x-x_{k}\right)=0, \end{array}$$

yielding a novel Newton update:

(9) $$\begin{array}{c} x_{k+1}=x_{k}-{\left(B_{k}+\frac{\rho }{2}\left\|x_{k}-x_{k-1}\right\|\cdot I\right)}^{-1}g_{k}, \end{array}$$

where *I* represents the identity matrix with the same size as **B**_*k*_. Comparing (5) with (9) additionally makes use of the norm of difference between previous two estimates, leading to better performance since it captures more curvature information.

### 2.3. Updating **B**_*k*_

The stochastic Hessian **B**_*k*_ can be updated based on the weak secant equation [40, 41]:

(10) $$\begin{array}{c} B_{k}=\underset{B}{\arg\min}\left\|B-B_{k-1}\right\|,\\ \text{s.t. }s_{k}^{T}Bs_{k}=s_{k}^{T}y_{k}\left(\text{weak secant equation}\right), \end{array}$$

where **s**_*k*_=**x**_*k*_ − **x**_*k*−1_ and **y**_*k*_=**g**_*k*_ − **g**_*k*−1_. The solution of the above problem with Frobenius matrix based on the variational technique in [42] is given by

(11) $$\begin{array}{c} B_{k}=B_{k-1}+\frac{s_{k}^{T}y_{k}-s_{k}^{T}B_{k-1}s_{k}}{{\left\|s_{k}\right\|}_{4}^{4}+\varepsilon }\text{Diag}\left(s_{k}^{2}\right), \end{array}$$

where Diag(**v**) is the diagonal matrix with diagonal elements from vector **v**. Further, with rectifying operation which guarantees the positive-definiteness, the updated cubic Newton becomes

(12) $$\begin{array}{c} x_{k+1}=x_{k}-D_{k}^{-1}g_{k}, \end{array}$$

where

(13) $$\begin{array}{c} D_{k}=\max\left(\mathrm{abs}\left(B_{k}+\frac{\rho }{2}\left\|x_{k}-x_{k-1}\right\|\cdot I\right),\theta \cdot I\right), \end{array}$$

where *θ* is a positive parameter, and the cost of computing **D** is marginal since **B**_*k*_ is diagonal, abs(**V**) takes absolute values of all the elements of the matrix **V**. It is worth mentioning that, according to equations (5) and (12), max(·, ·) operation enables **D**_*k*_ to prevent the step size from becoming arbitrary large since there exists zero value in **B**_*k*_.

### 2.4. Moments for **g**_*k*_ and **D**_*k*_

In this paper, we adopt the moments for **g**_*k*_ and **D**_*k*_, given by

(14) $$\begin{array}{c} m_{k}⟵\beta_{1}m_{k-1}+\left(1-\beta_{1}\right)g_{k},\\ V_{k}⟵\beta_{2}V_{k-1}+\left(1-\beta_{2}\right)D_{k}⊙D_{k}, \end{array}$$

where ⊙ denotes the elementwise multiplication, and *β*_1_, *β*_2_ ∈ (0,1) are the first and second moment hyperparameters that are also used in Adam [8] and its many variants. The moments are further bias corrected as

(15) $$\begin{array}{c} {\hat{m}}_{k}⟵\frac{m_{k}}{\left(1-\beta_{1}^{k}\right)},\\ {\hat{V}}_{k}⟵\frac{V_{k}}{\left(1-\beta_{2}^{k}\right)}. \end{array}$$

Using the first and second moment amounts to carrying out an exponential moving average on iteratively updated stochastic gradients and approximated stochastic Hessians plus the norm of difference between previous two estimates, which can smooth the noisy curvature information and get an approximation to the global curvature information, avoiding misleading local gradient and Hessian information which can be catastrophic.

To summarize, the complete algorithm of AdaCN is given in Algorithm 1, in which at most first order gradients are required, and **B**_*k*_, **D**_*k*_, **V**_*k*_, and ${\hat{V}}_{k}$ are all diagonal. Therefore, AdaCN updates with linear complexity for both time and memory.

## 3. Experiments

In this section, we access the performance of AdaCN on learning tasks: image classification and language modeling, comparing with stochastic first order optimizers such as Adam [8], SGD [1], AdaBound [13], and stochastic second order optimizer Apollo [20], listed in Table 1. For image classification, we investigate models by LeNet [31] on Mnist and VGG11 [32], ResNet34, and DenseNet121 [34] on CIFAR10 and CIFAR100 [35], while for language modeling, LSTM [36] on Penn Treebank [37] is tested. Moreover, the robustness to hyperparameters is tested, through comparing AdaCN and Apollo with different values of *ε* and learning rate. The results are shown in the following subsections.

### 3.1. Experiments Setup

We perform a careful hyperparameter tuning in experiments as follows. AdaCN: we set *θ*=1, *β*_1_=0.9, *β*_2_=0.999, *ε*=10^−8^, and *ρ*=5 × 0.9^200−*k*^ at *k*-th iteration. The learning rate *η*=0.4 for Mnist dataset, 0.2 for CIFAR datasets, and 30 for Penn Treebank dataset. SGD: the momentum is set to 0.9, while the learning rate is searched among {*a* × 10^*b*^} where *a* ∈ {1,2,3,4,5,6,7,8,9} and *b* ∈ {−3, −2, −1,0,1}. Adam, AdaBound, and Apollo: the learning rate is searched as SGD, and other parameters are set as their own default values in the literature.

### 3.2. Image Classification

At first, we evaluate the convergence and generalization of AdaCN on image classification. We use LeNet on Mnist and VGG11, ResNet34, and DenseNet121 on CIFAR10 and CIFAR100 dataset.

*Mnist*. Results on Mnist are shown as Figure 2: the curves of train and test accuracy on Mnist and Table 2, from which we can see that AdaCN achieves the best convergence speed and classification accuracy.

*CIFAR10*. We report the results on CIFAR10 in Figure 3 and Table 3. For all three network architectures, AdaCN obviously outperforms other optimizers with comparable convergence speed and best classification accuracy.

*CIFAR100*. Results on CIFAR100 are shown in Figure 4 and Table 4. For VGG11, AdaCN is better than Adam and Apollo, but worse than SGD and AdaBound in terms of convergence speed and classification accuracy. For ResNet34 and DenseNet121, AdaCN achieves the best classification accuracy.

### 3.3. Language Modeling

On language modeling, we experiment with 1, 2, 3-layer LSTM model on Penn Treebank dataset. As Figure 5 and Table 5 show, AdaCN can also keep fastest convergence speed and achieve the lowest perplexity among the optimizers for 1, 2, 3-layer LSTM.

Finally, we explore the effects of the hyperparameters including *ε* and learning rates on the performance of AdaCN, respectively. The results on CIFAR10 dataset are reported in Figures 6 and 7, where the values of *ε* are ranging from 10^−3^ to 10^−7^ in a log-scale grid on ResNet34 and learning rate ranging from 5 × 10^−3^ to 2 × 10^−1^ on VGG11, respectively. As can be seen, the test accuracies of AdaCN are above 95% for all values of *ε*, while Apollo achieves an accuracy consistently below 95%. Moreover, the results validate the robustness of AdaCN to *ε* and learning rate.

## 4. Conclusion

We have proposed AdaCN, a novel, efficient, and effective adaptive cubic Newton method for nonconvex stochastic optimization. This method is designed for large-scale nonconvex stochastic optimization problems which are the core of state-of-the-art deep learning literature. Experimental results on image classification tasks and language modeling task demonstrate the superiority of AdaCN, in terms of convergence speed and generalization performance.

## Figures and Tables

**Figure 1:** Trajectories of SGD, Adam, Apollo, and AdaCN on a convex function (a) and a nonconvex function (b), respectively. Parameters of two experiments are set as follows: the learning rates of AdaCN, Apollo, Adam, and SGD are set to 2 × 10^−3^, 2 × 10^−3^, 3 × 10^−2^, and 5 × 10^−4^, respectively. For SGD and Apollo, *β*=0.9, whereas for AdaCN and Adam, *β*_1_=0.9 and *β*_2_=0.9. The model is trained for 2.5 × 10^3^ epochs. (a) Loss function is *f*(*x*, *y*)=(*x*+*y*)^2^+(*x* − *y*)^2^/10. (b)*f*(*x*, *y*)=(*x* − 1)^2^+100(*y* − *x*^2^)^2^.

**Figure 2:** The curves of train and test accuracy on Mnist. (a) Train Accuracy. (b) Test Accuracy.

**Figure 3:** The curves of train and test accuracy on CIFAR10. (a) Train accuracy of VGG11 on CIFAR10. (b) Test accuracy of VGG11 on CIFAR10. (c) Train accuracy of ResNet34 on CIFAR10. (d) Test accuracy of ResNet34 on CIFAR10. (e) Train accuracy of DenseNet121 on CIFAR10. (f) Test accuracy of DenseNet121 on CIFAR10.

**Figure 4:** The curves of train and test accuracy on CIFAR100. (a) Train accuracy of VGG11 on CIFAR100. (b) Test accuracy of VGG11 on CIFAR100. (c) Train accuracy of ResNet34 on CIFAR100. (d) Test accuracy of ResNet34 on CIFAR100. (e) Train accuracy of DenseNet121 on CIFAR100. (f) Test accuracy of DenseNet121 on CIFAR100.

**Figure 5:** The curves of test perplexity on Penn Treebank for 1, 2, 3-layer LSTM. Lower is better. (a) Test perplexity for 1-layer LSTM. (b) Test perplexity for 2-layer LSTM. (c) Test perplexity for 3-layer LSTM.

**Figure 6:** The curves of train and test accuracy of ResNet34 on CIFAR10 with respect to different values of *ε*. (a) Train accuracy of AdaCN on CIFAR10. (b) Train accuracy of Apollo on CIFAR10. (c) Test accuracy of AdaCN on CIFAR10. (d) Test accuracy of Apollo on CIFAR10.

**Figure 7:** The curves of train and test accuracy of VGG11 on CIFAR10 with respect to different values of learning rate. As can be seen, AdaCN is more robust to learning rate. (a) Train accuracy of AdaCN on CIFAR10. (b) Train accuracy of Apollo on CIFAR10. (c) Test accuracy of AdaCN on CIFAR10. (d) Test accuracy of Apollo on CIFAR10.

**Algorithm 1:** AdaCN.

**Table 1:** Summaries of the settings used in experiments.

Task	Dataset	Network type	Architecture	Optimizer
Image classification	Mnist	Convolutional neural network	LeNet	AdaCN, Apollo, Adam, SGD, AdaBound
	CIFAR10 CIFAR100		VGG11, ResNet34, DenseNet121	
Language modeling	Penn Treebank	Recurrent	1, 2, 3-layer LSTM	

**Table 2:** Test accuracy of LeNet on Mnist.

Model	Adam	SGD	AdaBound	Apollo	AdaCN
LeNet	0.984	0.981	0.987	0.988	**0.989**

The best result is shown in bold.

**Table 3:** Test accuracy of VGG11, ResNet34, and DenseNet121 on CIFAR10.

Model	Adam	SGD	AdaBound	Apollo	AdaCN
VGG11	88.40	89.72	90.60	88.90	**91.34**
ResNet34	93.02	93.62	94.75	94.79	**95.15**
DenseNet121	92.79	93.07	94.58	94.85	**95.52**

The best results are shown in bold.

**Table 4:** Test accuracy of VGG11, ResNet34, and DenseNet121 on CIFAR100.

Model	Adam	SGD	AdaBound	Apollo	AdaCN
VGG11	58.96	**66.01**	65.92	58.50	65.51
ResNet34	71.39	76.98	76.88	76.42	**77.11**
DenseNet121	71.85	79.35	79.00	79.01	**79.50**

The best results are shown in bold.

**Table 5:** Test accuracy of 1, 2, 3-layer LSTM on Penn Treebank dataset.

Model	Adam	SGD	AdaBound	Apollo	AdaCN
1-layer LSTM	86.86	86.14	85.68	84.90	**83.40**
2-layer LSTM	68.81	68.54	68.58	69.71	**68.17**
3-layer LSTM	64.91	64.50	65.18	66.37	**63.26**

The best results are shown in bold.

## Data Availability

The data used to support the findings of this study are open datasets which could be found in general websites, and the datasets are also freely available.
